# Determination of Wheat Heading Stage Using Convolutional Neural Networks on Multispectral UAV Imaging Data

**DOI:** 10.1155/2022/3655804

**Published:** 2022-11-24

**Authors:** Yibai Li, Guangqiao Cao, Dong Liu, Jinlong Zhang, Liang Li, Cong Chen

**Affiliations:** Nanjing Institute of Agricultural Mechanization, Ministry of Agriculture and Rural Affairs, Nanjing 210014, China

## Abstract

The heading and flowering stages are crucial for wheat growth and should be used for fusarium head blight (FHB) and other plant prevention operations. Rapid and accurate monitoring of wheat growth in hilly areas is critical for determining plant protection operations and strategies. Currently, the operation time for FHB prevention and plant protection is primarily determined by manual tour inspection of plant growth, which has the disadvantages of low information gathering and subjectivity. In this study, an unmanned aerial vehicle (UAV) equipped with a multispectral camera was used to collect wheat canopy multispectral images and heading rate information during the heading and flowering stages in order to develop a method for detecting the appropriate time for preventive control of FHB. A 1D convolutional neural network + decision tree model (1D CNN + DT) was designed. All the multispectral information was input into the model for feature extraction and result regression. The regression revealed that the coefficient of determination (*R*^2^) between multispectral information in the wheat canopy and the heading rate was 0.95, and the root mean square error of prediction (RMSE) was 0.24. This result was superior to that obtained by directly inputting multispectral data into neural networks (NN) or by inputting multispectral data into NN via traditional VI calculation, support vector machines regression (SVR), or decision tree (DT). On the basis of FHB prevention and control production guidelines and field research results, a discrimination model for FHB prevention and plant protection operation time was developed. After the output values of the regression model were input into the discrimination model, a 97.50% precision was obtained. The method proposed in this study can efficiently monitor the growth status of wheat during the heading and flowering stages and provide crop growth information for determining the timing and strategy of FHB prevention and plant protection operations.

## 1. Introduction

Wheat is an essential food crop, and ensuring its yield and quality is critical to food safety [1, 2] Fusarium head blight (FHB) is a major wheat disease that affects global wheat yield [3, 4]. According to the 2016 Technical Guidelines on the Preventive Control of FHB issued by the Ministry of Agriculture and Rural Development (MARD) and the general concept of “prevention first” when it comes to related agronomic requirements, preventive control should be applied to FHB because it is highly infectious, is difficult to cure [5, 6], and significantly impacts yield [7–9]; Similar control should also be applied to other pests and diseases [10, 11], such as aphids and powdery mildew [12, 13], respectively. The guidelines state that the best time to prevent and control FHB is from the flush to the early flowering stages. The timing of pesticide spraying has a significant impact on disease prevention, and the time required to control FHB is highly connected with the wheat heading rate [14]. In practice, monitoring wheat heading rates is primarily achieved through manual tour inspection, which is inefficient and subjective. Thus, quickly and accurately determining the wheat heading rate is critical for the preventive control effect of FHB [15]. In addition, studies and experiments have demonstrated that mastering the crop operation time window is important for planning the operation strategy of plant protection machinery and improving the effectiveness and efficiency of plant protection operations [16, 17].

Current studies on monitoring the developmental stages of wheat mainly focus on the tillering, flowering, and grain filling stages, with wheat chlorophyll, leaf area index (LAI), etc., as the monitoring targets [18, 19]. There are also some studies that focused on the monitoring of FHB after its onset [20]. However, studies on the monitoring of the FHB prevention operation period during the heading and flowering stages are scarce. Low-altitude remote sensing technology based on an unmanned aerial vehicle (UAV) has been used in monitoring crop growth owing to its advantages of high mobility, simplicity, and safety [21]. Multispectral cameras can acquire information at more wavelengths than ordinary digital ones and have a lower price than hyperspectral ones. This hardware is more advantageous in terms of monitoring effects and cost-efficiency [22]. Common multispectral information processing methods include neural networks (NN), support vector machines (SVM), decision trees (DT), and other simple feature extraction methods, all of which can achieve relatively good target fitting accuracy [23–25]. Previous experimental processes with chlorophyll, leaf area, and nitrogen changes as research objectives had long data acquisition intervals, with relatively great changes in crop growth states. Hence, they were less demanding on the feature extraction capacity of fitting models. During the heading and flowering stages, wheat has no evident changes in features other than the heading rate, which rapidly changes. Thus, better feature extraction and expression capacity of the regression model are required [26–28]. Convolutional neural network (CNN) has a high capacity for feature extraction and expression and has been widely used in image processing, video analysis, and other fields [29–31]. In addition, CNN has been applied to spectral analysis. Convolutional kernels are used as filters in CNN to extract multilevel features of information by superimposing multiple layers of convolutional kernels [32, 33]. The convolutional neural network requires a large number of samples to train the weights of the convolution kernels. The number and dimensions of the convolution kernels have different requirements for the number of training samples [34]. The more the number of convolution kernels, the higher the dimension of the convolution kernels. The lack of training data or the high cost of obtaining training data is the biggest obstacle to the failure of convolutional neural network fitting to play a good role in different scenarios [35]. Thus, the method can extract complex features from high-dimensional data. In the processing of one-dimensional information such as text and speech, 1D CNN also exhibits good performance [36, 37]. Due to the low dimension of the convolution kernel, the 1D CNN has a good performance in the field of text and language processing with small training samples [38]. In the field of crop growth state exploration, studies have shown that can have a better fitting effect on the processing of small samples of crop spectral information [39]. Under the same network structure, 1D CNN has some advantages, the number of link weights is smaller than that of 2D CNN, the number of training samples required is much smaller than the 2D CNN. Therefore, this study proposed the extraction of wheat spectral features by 1D CNN to address the problem of wheat heading rate fitting during the heading and flowering stages.

In summary, to solve the problem of low efficiency and subjectivity in information acquisition for determining the operation time of FHB prevention and plant protection in hilly areas, this study proposed the collection of spectral information of wheat canopy during the heading and flowering stages using a UAV equipped with a multispectral camera and designing a 1D CNN + DT model to extract the spectral information and fit the wheat heading rate. On this basis, a 1D CNN structure was designed for feature extraction of spectral information. Then, the features extracted by the fully connected layer were input into the decision tree (DT) to fit the earing rate to improve the regression effect of the model. According to the requirements of FHB prevention and plant protection time, a discrimination model for FHB prevention and plant protection operations was established to provide a crop state fast discriminative method for determining the unified prevention and control time and intelligent plant protection equipment operation strategy during the wheat heading stage.

## 2. Materials and Methods

Experimental data were collected in Taiping Village, Xixia District, Nanjing, Jiangsu Province. Taiping Village is located northeast of Nanjing and downstream of the Yangtze River. The experimental area has a plain terrain, a humid north subtropical climate, four distinct seasons, rain and heat in the same season, abundant sunshine, an average annual precipitation of 1,090.4 mm, an average annual temperature of 15.4°C, and a frost-free period of 237 days. The soil type is yellow brown loam. In this paper, the wheat varieties collected were Zhenmai 7, Yangmai 12, and Yangmai 16, with one plot per variety, about 0.3 ha per plot. The collection period was performed daily from April 11 to April 20, 2021, covering the states of 0% to 100% head emergence.

### 2.1. Data Acquisition and Preprocessing

#### 2.1.1. Multispectral Data Acquisition

In this study, remote sensing data on wheat canopy were collected using a 10 kg XAG XMISSION UAV with a maximum load of 6 kg. The target plot was selected in the smartphone system, and the UAV flew according to the route trajectory automatically planned by the system at a height and speed of 9 m and 3 m/s, respectively. The 0.85 kg multispectral camera had 20 million pixels and an image resolution of 3863 × 3648 pixels, covering four bands, the wavelengths of 550, 660, 735, and 790 nm for the corresponding central bands with 20 megapixels. The standard whiteboard (50 × 50 cm) was placed in each experimental plot as the radiation correction data for the later remote sensing data.

#### 2.1.2. Processing of Multispectral Data

After the acquisition, the data from the UAV hyperspectral remote sensing needed to be processed, and the data processing procedure was divided into two parts: (1) extraction of the region of interest (ROI) from multispectral images by manually extracting a rectangular box (50 × 50 pixels) and averaging the values within the ROI as sample data. (2) Radiation correction by calibrating the location of the standard whiteboard with a rectangle box (3030 pixels) and averaging the values as the white standard correction value. On this basis, radiation correction CI is achieved using equation (1), where *W* denotes the spectral mean of the standard whiteboard in the band on that day; *I*, the spectral mean of the samples in the band on that day; and *B*, the pixel mean in the band when the lens is covered.

(1) $$\begin{array}{c} CI=\frac{I-B}{W-B}\text{.} \end{array}$$

In addition to inputting the information of each wavelength band directly into the fitting model, the transformation of every two or more band values into vegetation index (VI) should also be investigated to highlight the crop characteristic changes and fit the target better. Based on the spectral wavelength values collected, the difference index (DI), difference vegetation index (DVI), red-edge chlorophyll index (CI_rededge_), normalized difference vegetation index (NDVI), green normalized difference vegetation index (GNDVI), and triangular vegetation index (TVI) [36] were selected. The information from the five vegetation indices above was used to fit the wheat heading rate. The indices are calculated using Equations (2)–(7), where *R* denotes the spectrum, and the subscript numbers represent the band of a specified wavelength. As the spectral resolution error of the spectrum instrument is ±30 nm, *R*_800_ can be replaced by the 790 nm band, *R*_680_ and *R*_670_ by the 660 nm band, and *R*_720_ and *R*_750_ by the 730 nm band.

(2) $$\begin{array}{c} DI=R_{800}-R_{550}\text{,} \end{array}$$

(3) $$\begin{array}{c} DVI=R_{800}-R_{680}\text{,} \end{array}$$

(4) $$\begin{array}{c} NDVI=\frac{\left(R_{780}-R_{670}\right)}{\left(R_{780}+R_{670}\right)}\text{,} \end{array}$$

(5) $$\begin{array}{c} {CI}_{re\;de\;dg\;t}=\left(\frac{R_{800}}{R_{720}}\right)-1\text{,} \end{array}$$

(6) $$\begin{array}{c} GNDVI=\frac{\left(R_{800}-R_{550}\right)}{\left(R_{800}+R_{550}\right)}\text{,} \end{array}$$

(7) $$\begin{array}{c} TVI=0.5*\left(120*\left(R_{750}-R_{550}\right)-200*\left(R_{670}-R_{550}\right)\right)\text{.} \end{array}$$

#### 2.1.3. Acquisition of Wheat Heading Rate Data

In this study, data for three wheat varieties were collected, with one plot for each variety and three random sampling sites randomly selected in each plot. The label data of each area was the wheat heading rate. The counting method was used to collect ear emergence rate data. Three marked areas were randomly selected for each plot, and each area contained *X* wheat plants. For the convenience of calculation, the *X* of each small area was 20. Statistic *A* was carried out on the wheat plants with ears emerging every day, and the percentage of wheat ears emerging in this area was calculated by the following equation:

(8) $$\begin{array}{c} X=\frac{A}{20}\text{.} \end{array}$$

### 2.2. Fitting Method

In the experiment, a total of 720 entries of multispectral data and corresponding heading rate labels were obtained; among them, 120 entries were randomly selected as test data, and the remaining 600 entries were used as training data.

#### 2.2.1. 1D CNN + DT Fitting Method

The minor changes in crop state during the wheat heading and flowering stage require higher feature extraction and expression capacity from 1D CNN. In the first few layers of 1D CNN, the surface features of information, such as color and texture, can be extracted; in the depth layers, the abstract features of information can be extracted. Better feature extraction functions can be obtained by stacking multiple layers. Based on this principle, this study designs the network structure by fusing the features extracted by the third layer with those extracted by the fifth layer and then inputting them into the fully connected layer. The convolutional kernels in the 1D CNN are all one-dimensional, and the convolutional kernel weights are initially determined using the random number method. As the input dimension is 4, the convolutional kernel has a size of 1 and a step size of 1. The “same” method is used to convolve the data. There are five convolutional layers in the NN, and the “LeakyReLu” function is used as the activation function in each layer. The dropout module is added to the last three layers to improve the training speed and generalization performance of the network, with the probability of dropout set to 0.1. The training objective function of 1D CNN adopts the mean squared logarithmic error with the formula presented in (9), where *n* denotes the number of data points in the whole dataset; *p*_*i*_, the predicted value; and *a*_*i*_ is the measured value. The weights of convolution kernels are optimized using the Adam method, where the learning rate is lr = 0.002, decay rat *e* = 1 *e* − 9, momentum = 0.5, and epoch = 1000.

(9) $$\begin{array}{c} \varepsilon =\frac{1}{n}\overset{n}{\underset{i=1}{\sum }}\left(\sqrt[{2}]{{\left(p_{i}-a_{i}\right)}^{2}}\right)\text{.} \end{array}$$

After the network is trained, based on the original network structure and convolution kernel weights. Input the data into the 1D CNN, extract the output in the fully connected layer as features, input the features into the decision tree (DT), use the decision tree to perform regression analysis on the feature information, and fit the wheat heading Rate. Equation (10) describes the training dataset for the decision tree. Assume that the output of the fully connected layer of the fully convolutional neural network is *fc*_*i*_, *DT* represents the predicted output value after the decision tree calculation, and *a*_*i*_ is the measured value. Decision tree generation Use ID3 for decision tree generation and C4.5 method for feature selection. In equations (11)–(13), the feature is *A*, and *H*(*D*) represents the empirical entropy of the dataset *D*. *H*(*D|A*) represents the empirical conditional entropy of feature *A* on the dataset, where *n* is the number of values taken for feature *A*. Equations (12) and (13) indicates the information gain ratio. In the input space where the training dataset is located, each region is recursively divided into two subregions.

(10) $$\begin{array}{c} \left.D=\left\{\left(DT\left({fc}_{1}\right),a_{1}\right)\right.,\left(DT\left({fc}_{2}\right),a_{2}\right),\ldots \left(DT\left({fc}_{i}\right),a_{i}\right)\right\}\text{,} \end{array}$$

(11) $$\begin{array}{c} g\left(D,A\right)=H\left(D\right)-H\left(\frac{D}{A}\right)\text{,} \end{array}$$

(12) $$\begin{array}{c} gr\left(D,A\right)=\frac{g\left(D,A\right)}{H_{A}\left(D\right)}\text{,} \end{array}$$

(13) $$\begin{array}{c} H_{A}\left(D\right)=-\overset{N}{\underset{n=1}{\sum }}\frac{\left|D_{i}\right|}{\left|D\right|}\log_{2}\left|\frac{D_{i}}{D}\right|\text{.} \end{array}$$

The 1D CNN + DT model structure is shown in Figure 1.

#### 2.2.2. NN, SVM, and DT Methods

In the neural network (NN), the nonlinear transformation method is employed to identify combinations of suitable parameters in the input and solution spaces to achieve the purpose of information transformation. Upon initialization of the network, connection weights between neurons at different levels are determined using the random number method, and the distance between the calculated and target values of the network is obtained using the minimum mean square error (MMSE) as the objective function. The error is propagated to each neuron's connection weight using the error backpropagation (BP) method, and the connection weights are adjusted according to the gradient descent direction and step size.

This study demonstrates that the ideal experimental structure is a 4-layer network with 4 neurons in the input layer, 30 neurons in the hidden layer, 15 neurons in the second hidden layer, and 1 neuron in the output layer. The neural network selected in this paper is shown in Figure 2.

A (Support Vector Machine Regression) SVR is a generalized linear classifier that performs binary classification of data in a supervised learning manner. Its boundary decision is to solve the maximum-margin hyperplane for the learned samples. As most data are nonlinearly differentiable, the kernel function approach is employed to map them into a high-dimensional space. In this study, the Gaussian kernel is used to translate the data into a high-dimensional space, and the MMSE is used to determine the SVM parameters by identifying the maximum-error partition plane.

A decision tree (DT) represents the conditional probability distribution of a given feature. From the training dataset, a set of classification or regression rules are inducted. The DT has a tree structure in which each node represents an object, each branch represents a possible attribute value, and each leaf node corresponds to the value of objects in the path from the root node to that leaf node. The nodes mainly include decision, chance, and end nodes. By pruning and learning, the tree structure with good fit and generalization performance is obtained.

Both NN and DT require iterations to determine the connection weights or tree structure. The number of iterations in this paper was 10,000.

Figure 3 is the working flow chart of this paper.

## 3. Experimental Results

### 3.1. Multispectral Reflectance and Heading Rates of Wheat

It can be seen from Figure 4 that the reflectance values of the 730 and 790 nm bands are larger than those of 550 and 660 nm, and the changing trends of the spectral reflectances of the four bands are different. In terms of varieties, Zhenmai 7 and Yangmai 16 have similar trends in each frequency band, and Yangmai 12 and the first two varieties are slightly different in individual days.

The changes in the heading rates of three varieties are presented in Figure 5, showing that Zhenmai 7 has a heading rate range of [0.08, 0.86], Yangmai 12 [0.27, 1], and Yangmai 16 [0.3, 1]. The heading rate variation trend of each variety is slightly different. The heading rate of Zhenmai 7 rapidly increases in the first 8 days and slowly from day eight to ten day; the heading rate of Yangmai 12 presents a rapid growth state in the first 3 days, with the heading rate rapidly increasing from 0.3 to 0.98, further growing from 0.98 to 1 during days 3–5, and remaining at 1 afterward; the heading rate of Yangmai 16 changes in the range of [0.3, 0.5] from day 1 to day 3 and [0.5, 1] from day 3 to day 8, with a moderate variation trend, and presents no more changes on days 9 and 10.

The variation trend of heading rates indicates that Zhenmai 7 and Yangmai 16 are similar, spanning 8 and 9 days from partial to full heading, whereas Zhenmai 12 has a high heading rate, spanning only 5 days from partial to full heading. The spectral change patterns of the three wheat varieties are compared. The results indicate that Zhenmai 7 and Yangmai 16 have a similar spectral change trend to Yangmai 12 and a similar heading rate trend to Yangmai 12. As a result, it can be concluded that there is a correlation between wheat multispectral information about the wheat canopy and heading rate.

### 3.2. Fitting Models of Wheat Heading Rate at Different Wavelengths

First, the single-band information is input into the fitting model based on 1D CNN + DT, neural network (NN), support vector machine (SVR) and decision tree (DT). The fitting result of the model is shown in Table 1.

It can be seen from the fitting effect that the fitting degree of each band is not high, and the highest fitting *R*^2^ does not exceed 0.6. In each band, the fitting degree of the 660 nm and 730 nm bands is higher, and the fitting degree of the 550 nm and 790 nm bands is slightly weaker. From the method point of view, the fitting degree of the 1D CNN + DT method is better than that of DT, and both outperform support vector machine and neural network.

### 3.3. Vegetation Index for Estimating Wheat Heading Rate

Regression is performed on the DI, DVI, CI_rededge_, NDVI, GNDVI, TVI, and wheat heading rate. The regression models adopt NN, SVM, and DT. The regression results are presented in Table 2.

#### 3.3.1. Regression Effect Analysis

TVI outperforms all other variables in terms of VI, with an *R*^2^ of 0.85, followed by CI_rededge_. TVI has an *R*^2^ of 0.76. TVI is calculated by weighting the information from three bands, which involves the red edge, red light, and green light; CI_rededge_ is mainly calculated by the red edge and infrared band. In terms of the methods, DT has better performance than SVM and NN in general, except that in CI_rededge_, SVM performs better than DT, and in *R*^2^, DT is 0.04 lower than SVM. However, its performance is still inferior to the 1D CNN + DT method, which indicates that CNN has excellent feature extraction capacity.

### 3.4. Fitting Models of Wheat Heading Rate at Different Wavelengths Combination

On this basis, all bands and multiple band combinations were used to fit the information of wheat ear emergence rate. The fitting model still chooses a neural network, support vector machine, decision tree, 1D CNN + DT. The performance of each band combination is shown in Table 3.

From the fitting effect of each band group, it can be seen that the fitting effect of the 550 + 660+730 + 790 nm band is the best, and the fitting effect of the band combination of 550 + 660 + 790 nm and 550 + 730 + 790 nm ranks first. The combination of 660 + 730 + 790 nm lacking the 550 nm band has the worst fitting effect. From the method point of view, the performance of 1D CNN + DT is the best, the performance of the decision tree method is second, and the performance of the neural network is the worst. To sum up, CNN has a stronger feature extraction ability than other methods. After extracting the features, it can be combined with the decision tree for regression analysis to obtain a better fitting effect. The convergence of all band combinations input into the 1D CNN + DT model is shown in Figure 6.

The predicted and measured values of wheat heading rate in multispectral prediction using the 1D CNN + DT method are presented in Figure 7. The figure shows that, on average, the predicted and measured values fit well, with discrepancies of less than 0.1; however, for a few data, the fit difference is 0.5 or greater. In practical applications, the influence of individual prediction errors on the accuracy of results can be reduced by selecting multiple ROIs on a remote sensing image.

It can be seen from the above-given results that the band combination of 550 + 660 + 730 + 790 nm and the 1D CNN + DT had good prediction ability for wheat heading emergence. In order to verify the feature extraction ability of 1D CNN + DT, this paper uses 400 pieces of 550 + 660 + 730 + 790 nm spectral data of all the data of Zhenmai 16 as the training data of 1D CNN + DT. 100 pieces of 550 + 660 + 730 + 790 nm spectral data of Yangmai 7 were used as test data to verify the accuracy of this method in predicting wheat heading emergence rate. The results show that the fitting coefficient *R*^2^ of the fitted model is 0.67, and the RMSEP of the fitting result is 0.32. The decision tree method with a better fitting effect among the above methods was used to fit the wheat spectrum to the ear emergence rate. The fitted correlation coefficient *R*^2^ was 0.47 and the RMESP was 0.48. It can be seen from the results that the monetization effect of the1D CNN + DT method in the new data set is somewhat lower than that of the old data set. At the same time, the decision tree performed worse on the new dataset. It shows that the generalization ability of such supervised algorithms is limited, and the spectral characteristics of different varieties of wheat are different. Comparing the two methods, the result of 1D CNN + DT is still better than that of a decision tree, which shows the effectiveness of this method.

### 3.5. Discrimination of Plant Protection Operation Time for Wheat FHB Prevention Based on Different Fitting Models

In this study, pursuant to the regulations on the application time in the 2016 Technical Guidelines on the Preventive Control of FHB issued by the MARD of the People's Republic of China, the period from wheat heading to early flowering is optimal for the prevention and control of the occurrence of FHB damage; “application upon flowering” can obtain twice the result with half the effort. When combined with the farmer experience, the period when the heading rate of the whole field reached 0.9 and above was determined to be the FHB preventive control operation period.

For the purpose of determining the significance and effectiveness of wheat heading rate monitoring in this paper, the combined waveband data or vegetation index were input into different monitoring models Determine whether the wheat is in the prevention and control period according to the output of the fitted model; that is, when the output value of the fitted model is greater than 0.9, it is determined that the wheat is in the prevention and control period. On the contrary, when the output of the fitted model is less than 0.9, the wheat is not in the prevention and control period. The discriminant accuracy of the final statistical fitting model.  Table 4 lists the discriminative accuracy rates of different band combinations or vegetation indices through different fitting models.

As presented in Table 4, the 1D CNN + DT model is superior to other methods for monitoring wheat heading rate, suggesting that CNN has a greater potential for feature extraction. Among the other methods, both DT and SVM have better judgment accuracy. In general, the DT has higher prediction accuracy. In terms of input bands, the fitting effect of full-band input has better prediction accuracy than other band combinations or traditional vegetation index methods. The band combination lacking 660 + 730 + 790 nm in other band combinations has the worst performance among all fitting models, which has a positive correlation with the fitting effect of the fitting model. In the traditional VIs, TVI has better prediction accuracy than the other indices as the other traditional VIs contain only two bands of information [as presented in equations (2)–(6), whereas TVI contains three bands [as presented in (7)]. However, the prediction accuracy of the fitting model established using the same method is lower than that with full-band information input, showing that better prediction accuracy can be obtained with full-band information for topping time determination.

In summary, a UAV was used to collect multispectral information on wheat, combined waveband information was selected, and a fitting model for the heading rate was established using the 1D CNN + DT method. The topping time was determined using the output of the fitting model, with an accuracy of up to 97.50%, and the optimal fitting effect was obtained.

## 4. Discussion

In this study, wheat canopy information was collected using UAV remote sensing technology. The heading rate fitting model was established to obtain the heading situation of wheat timely and rapidly and provide basic information on the crop for determining the operational time for unified prevention and control of FHB.

Multiple studies have established that UAV-based multispectral remote sensing technology is capable of monitoring quality-related characteristic indices such as nitrogen, chlorophyll, and LAI of wheat in real time. In terms of band information, the analysis results in this paper indicated that the use of combined bands of 550, 660, 730, and 790 nm had a better fit than the other VIs involving two or three bands. Studies by Wei et al. [30] and Yingxue et al. [31] demonstrated that the near-infrared and red-edge regions had a good effect on wheat nitrogen detection; studies by Shuangli et al. [32], Haojie et al. [33], and Feng et al. [34] demonstrated that the sensitive band for wheat chlorophyll prediction was the red-edge band. The sensitive wavebands of the wheat LAI were orange light and the red range; the use of orange light, red edge, and near-infrared wavebands to monitor wheat growth status had relatively good results, similar to the conclusions for heading rate monitoring in this study. Wheat heading rate and wheat growth status are closely related, and the comprehensive use of visible and infrared information bands can better monitor the growth status of wheat.

In terms of methods, CNN outperforms other methods in image recognition and segmentation. This is because CNN transforms the input data into a nonlinear space using convolution and activation functions and extracts the surface and deep features of the data via multilayer convolutional kernel transformation, which extracts more deep semantic features and thus presents the results more effectively. In terms of wheat growth state monitoring, studies by Bao et al. [35] and Qiu et al. [36] used CNN to monitor the diseases during the growth of wheat. The monitoring results indicated that the deep learning approach was superior to the other methods in feature extraction, disease identification, and monitoring capacity, which was consistent with the findings of this study. In terms of 1D CNNs, a study by Qin et al. [37] used 1D CNN to identify and classify the electrical signals of plants, with the accuracy improved by 7.7% compared with the classification accuracy of principal component analysis, leading to the conclusion that 1D CNN had better performance than the other models in this study. In terms of spectral analysis, studies by Zhao et al. [38] and Ma et al. [39] used 1D CNN to analyze Raman spectra. The analysis results indicated that 1D CNN + DT had better processing results than SVR, NN, and other methods. This is similar to the results of this study, which showed that in multispectral information processing, 1D CNN + DT still had a greater analytical advantage.

## 5. Conclusions

1. The combination of 550 + 660 + 730 + 790 nm bands fits the wheat heading rate better than the traditional VI.
2. A 1D CNN + DT structure was designed to process wheat canopy spectral information, and the fitting correlation coefficient between canopy multispectral data and the heading rate processed by the fitting model could reach 0.95 with an RMSEP of 0.24. The prediction results were 97.50% correct in determining the unified preventive control time for FHB.

The data collection and processing model in this study can provide crop data support for the determination of the unified preventive control time and strategy during the wheat heading stage.

## Figures and Tables

**Figure 1:** 1D CNN + DT model structure.

**Figure 2:** Diagram of neural network structure.

**Figure 3:** Multispectral information acquisition equipment and process.

**Figure 4:** Diagram of wheat spectral reflectance at different wavelength bands. (a) 550 nm. (b) 660 nm. (c) 730 nm. (d) 790 nm.

**Figure 5:** Diagram of heading rate variations of multiple wheat varieties.

**Figure 6:** 1D CNN + DT model training convergence process.

**Figure 7:** Fitting test plot of wheat heading rate based on the CNN fitting method.

**Table 1:** Fitting effect of single band information input fitting model.

Input band (nm)	Fitting model	Fitting results	
		*R* ^2^	RMSEP
550	NN	0.13	0.12
	SVR	0.12	0.07
	DT	0.36	0.39
	1D CNN + DT	0.47	0.37

660	NN	0.10	0.10
	SVR	0.11	0.10
	DT	0.46	0.38
	1D CNN + DT	0.57	0.39

730	NN	0.15	0.12
	SVR	0.26	0.17
	DT	0.47	0.40
	1D CNN + DT	0.52	0.37

790	NN	0.13	0.12
	SVR	0.27	0.17
	DT	0.40	0.32
	1D CNN + DT	0.47	0.34

**Table 2:** Fitting effect of traditional VI and heading rate.

Index	Method	Fitting result	
		*R* ^2^	RMSE
DI	NN	0.23	0.15
	SVM	0.40	0.20
	DT	0.55	0.31
	1D CNN + DT	0.57	0.31

DVI	NN	0.26	0.16
	SVM	0.28	0.17
	DT	0.63	0.35
	1D CNN + DT	0.70	0.36

NDVI	NN	0.27	0.17
	SVM	0.44	0.22
	DT	0.64	0.39
	1D CNN + DT	0.66	0.39

CI_rededge_	NN	0.23	0.15
	SVM	0.76	0.32
	DT	0.72	0.36
	1D CNN + DT	0.74	0.37

GNDVI	NN	0.27	0.17
	SVM	0.42	0.21
	DT	0.60	0.36
	1D CNN + DT	0.62	0.36

TVI	NN	0.13	0.31
	SVM	0.78	0.29
	DT	0.85	0.41
	1D CNN + DT	0.87	0.42

**Table 3:** Fitting effect of each band combination input fitting model.

Input band (nm)	Fitting model	Fitting results	
		*R* ^2^	RMSEP
550 + 660 + 730 + 790 nm	NN	0.77	0.24
	SVR	0.78	0.29
	DT	0.83	0.25
	1D CNN + DT	0.95	0.24

550 + 660 + 730 nm	NN	0.14	0.12
	SVR	0.58	0.25
	DT	0.76	0.24
	1D CNN + DT	0.82	0.24

550 + 660 + 790 nm	NN	0.12	0.48
	SVR	0.68	0.27
	DT	0.74	0.23
	1D CNN + DT	0.92	0.29

550 + 730 + 790 nm	NN	0.11	0.58
	SVR	0.69	0.27
	DT	0.70	0.26
	1D CNN + DT	0.92	0.28

660 + 730 + 790 nm	NN	0.11	0.43
	SVR	0.68	0.37
	DT	0.74	0.36
	1D CNN + DT	0.76	0.42

**Table 4:** Comparison of the accuracy of FHB preventive control time based on different monitoring models.

Monitoring model	Input band	Accuracy (%)
1D CNN + DT	550 + 660 + 730 + 790 nm	97.50
	550 + 660 + 730 nm	93.06
	550 + 660 + 790 nm	91.53
	550 + 730 + 790 nm	88.47
	660 + 730 + 790 nm	86.53
	DI	87.92
	DVI	91.39
	NDVI	89.72
	CI_rededge_	87.36
	GNDVI	87.36%
	TVI	89.36

NN	550 + 660 + 730 + 790 nm	67.22
	550 + 660 + 730 nm	67.22
	550 + 660 + 790 nm	67.22
	550 + 730 + 790 nm	63.75
	660 + 730 + 790 nm	56.94
	DI	56.94
	DVI	56.82
	NDVI	56.94
	CI_rededge_	59.17
	GNDVI	57.64
	TVI	63.33

SVM	550 + 660 + 730 + 790 nm	95.00
	DI	60.00
	550 + 660 + 730 nm	83.06
	550 + 660 + 790 nm	89.31
	550 + 730 + 790 nm	88.19
	660 + 730 + 790 nm	82.44
	DVI	71.81
	NDVI	72.22
	CI_rededge_	71.81
	GNDVI	60.97
	TVI	76.81

DT	550 + 660 + 730 + 790 nm	91.94
	DI	86.94
	550 + 660 + 730 nm	92.64
	550 + 660 + 790 nm	91.94
	550 + 730 + 790 nm	92.08
	660 + 730 + 790 nm	91.22
	DVI	89.17
	NDVI	88.33
	CI_rededge_	85.28
	GNDVI	89.17
	TVI	87.92

## Data Availability

The remote sensing data and codes used in the experiments to support the findings of this study are available from the corresponding author upon request.
